# An Automatic Knee Osteoarthritis Diagnosis Method Based on Deep Learning: Data from the Osteoarthritis Initiative

**DOI:** 10.1155/2021/5586529

**Published:** 2021-09-27

**Authors:** Yifan Wang, Xianan Wang, Tianning Gao, Le Du, Wei Liu

**Affiliations:** ^1^Department of Electrical Engineering, The University of Texas at Dallas, Richardson, TX, USA; ^2^National Clinical Research Center for Aging and Medicine, Huashan Hospital, Fudan University, Shanghai, China

## Abstract

Osteoarthritis (OA) is the most common form of arthritis. According to the evidence presented on both sides of the knee bones, radiologists assess the severity of OA based on the Kellgren–Lawrence (KL) grading system. Recently, computer-aided methods are proposed to improve the efficiency of OA diagnosis. However, the human interventions required by previous semiautomatic segmentation methods limit the application on large-scale datasets. Moreover, well-known CNN architectures applied to the OA severity assessment do not explore the relations between different local regions. In this work, by integrating the object detection model, YOLO, with the visual transformer into the diagnosis procedure, we reduce human intervention and provide an end-to-end approach to automatic osteoarthritis diagnosis. Our approach correctly segments 95.57% of data at the expense of training on 200 annotated images on a large dataset that contains more than 4500 samples. Furthermore, our classification result improves the accuracy by 2.5% compared to the traditional CNN architectures.

## 1. Introduction

Knee osteoarthritis (OA) is a significant reason for the disability of older people and the young. Recent research shows the knee OA will affect at least 130 million people by the year 2050, along with the globally aging population [1]. Treatment of knee OA has contributed more than 20 billion dollars in health expenditures [2]. Treatment options are limited for late-stage OA. Thus, it is crucial to detect and assess OA as early as possible to reduce the patient's suffering. While risk factors such as age and gender are helpful in the diagnosis of OA, medical imaging modalities are crucial in confirming and distinguishing OA from other forms of arthritis. Common image modalities include plain radiographic images (X-ray), ultrasound, and MRI [3]. X-ray is the most cost-efficient and convenient modality among the above three methods, accounting for a significant portion of clinical practice.

For several years, researchers studied X-ray analysis and diagnosis using computer-assisted methods. However, automatic OA severity assessment remains challenging for two reasons: (1) the lesion area occupies a small portion of the X-ray image. The irrelevant parts like clothes, tissues, or muscles overwhelm the cartilage status and mislead final decisions. (2) As bones differ in shape and density from one to another, it is challenging to establish standard diagnostic criteria. A well-trained radiologist assesses the severity of OA based on personal experiences, which are difficult to be incorporated into the computer-aided system.

Recent machine learning-based research introduced two stages shown in Figure 1 for automatic OA diagnosis: (1) the region of interest (ROI) segmentation, which suppresses noises by removing the background and irrelevant parts, and (2) the machine learning-based OA severity classification, which standardizes and simplifies complicated diagnostic criteria. However, previous knee detection methods depend on intensive human intervention to select features. In addition, OA symptoms may appear on different regions of the bone. The machine learning models applied for the OA diagnosis rarely explore the correlations of different regions, which undermines the assessment accuracy.

In this work, we followed the pipeline shown in Figure 1 but proposed an automatic procedure based on deep learning to assist the OA diagnosis on a large-scale dataset. Our main contributions are as follows:

1. We fine-tuned an object detection CNN to segment knees from X-ray images, which reduced the human interventions of feature engineering.
2. We exploited the self-attention mechanism by the visual transformer to improve the classification performance.
3. We examined the proposed method by classifying the OA severity based on the Kellgren and Lawrence (KL) level [4] over a large-scale dataset. The results show that the proposed method improves the efficiency of knee segmentation and the accuracy of OA severity classification.

This paper is organized as follows.  Section 2 reviews the previous work related to assisting the automatic OA diagnosis.  Section 3 presents the proposed approach in detail.  Section 4 shows the experiment results and discussions. Finally, Section 5 gives our conclusions.

## 2. Related Work

### 2.1. Knee Segmentation

Previous research on automatic OA assessments relies on manual or semiautomatic methods to segment knees. For example, [5] used a pattern match with 20 predetermined templates and [6] employed activate shape model (ASM), which picks bone texture features to guide analysis, whereas, in the human visual domain or the computer vision domain, knee segmentation requires prior knowledge. Human intervention, for example, tuning the parameters for the extracting algorithm, is inevitable when processing the new unseen samples. In the latter study [7], ROIs are proposed using a human-designed expert system guided by the sliding window. The author then uses a support vector machine (SVM) to determine the proper knee segmentation from the proposed regions. Overall, the introduction of machine learning methods improves the efficiency of knee segmentation tasks. However, human efforts are necessary to design an expert system and select background samples. As a result, it is difficult to apply the above methods to a large-scale dataset.

In recent years, object detection CNNs help with locating and recognizing ROIs in plain images. Well-known object detection networks include faster R-CNN [8], mask R-CNN [9], and YOLO [10]. A common technique shared by all three approaches is bounding box regression [8, 10], which handles the object's location and size separately. The bounding box is a rectangle which tightly covers one object. Each object's location and size are determined by the center coordinates of its bounding box, denoted as *x*_obj_, *y*_obj_, and the bounding box height and width, denoted as *h*_obj_, *w*_obj_. In general, CNNs do not directly predict location and size but retrieve them through a decoding process from the outputs. For example, the YOLO model relies on two additional information to decode its outputs for locations and sizes, respectively. For object locations, the authors of [10] introduced a reference grid system, which evenly divides the entire image into small squared regions. Each grid has corresponding outputs *x*_out_ and *y*_out_ from the YOLO model. The predicted object center coordinates *x*_pred_ and *y*_pred_ are retrieved from

(1) $$\begin{array}{c} \left\{\begin{array}{c} x_{\text{pred}}=\sigma \left(x_{\text{out}}\right)\times l_{\text{grid}}+x_{\text{grid}},\\ y_{\text{pred}}=\sigma \left(y_{\text{out}}\right)\times l_{\text{grid}}+y_{\text{grid}}, \end{array}\right. \end{array}$$

where *σ* is the sigmoid function, *l*_grid_ is the grid edge length, and *x*_grid_ and *y*_grid_ are the top left corner coordinates of one grid. As the sigmoid function in equation (1) restricts outputs to the range of (0,1), a grid only predicts the objects within the region. However, the YOLO model detects an object at an arbitrary location by applying equation (1) to all grids. Regarding object sizes, the YOLO outputs are decoded referring to the “anchors.” Anchors are the prior knowledge of the object size determined by clustering the sizes of all training objects. In practice, the YOLO model used cluster centroids as the expected shapes of an object. The outputs of YOLO, denoted as *w*_out_ and *h*_out_, calibrate the anchors to retrieve the predicted size *w*_pred_ and *h*_pred_ using

(2) $$\begin{array}{c} \left\{\begin{array}{c} w_{\text{pred}}=w_{\text{anchor}}\times \;\exp\left(w_{\text{out}}\right),\\ h_{\text{pred}}=h_{\text{anchor}}\times \;\exp\left(h_{\text{out}}\right), \end{array}\right. \end{array}$$

where *w*_anchor_ and *h*_anchor_ are the width and height of the anchor. With equations (1) and (2), the YOLO model solves the detection problem as a regression task. Equation (3) computes the regression errors as follows:

(3) $$\begin{array}{c} \left\{\begin{array}{c} x_{\text{err}}={\left(x_{\text{obj}}-x_{\text{pred}}\right)}^{2},\\ y_{\text{err}}={\left(y_{\text{obj}}-y_{\text{pred}}\right)}^{2},\\ w_{\text{err}}={\left(\sqrt{w_{\text{obj}}}-\sqrt{w_{\text{pred}}}\right)}^{2},\\ h_{\text{err}}={\left(\sqrt{h_{\text{obj}}}-\sqrt{h_{\text{pred}}}\right)}^{2}. \end{array}\right. \end{array}$$

Notably, the errors in equation (3) only account for the grids which contain ground truth object. To distinguish the objects from the background, the YOLO model is also trained by a confidence error as in

(4) $$\begin{array}{c} {\mathrm{conf}}_{\text{err}}={ℒ}_{\mathrm{BCE}}\left(\sigma \left(p_{\text{out}}\right),p_{\text{obj}}\right), \end{array}$$

where ℒ_BCE_ is the binary cross entropy loss function, *p*_out_ is the confidence output of each grid, and *p*_obj_ is an indicator of object existence. Particularly, if a grid covers at least one object center, the corresponding *p*_obj_ is set to 1. Otherwise, *p*_obj_ is set to be 0.

For our task, each knee joint's visual structure is clear, but its position and size are difficult to detect. Bounding box regression boosts segmentation performance and minimizes the human effort in designing a sophisticated extraction system.

### 2.2. Image Classification

In the light of deep learning, CNNs are becoming a prevalent image classification technique [11, 12]. Generally, a CNN consists of three sequential parts: convolutional layers for feature extraction, a pooling layer for spatial feature fusion, and one or two linear layers for the classification. Previous studies applied the CNNs to extract features from the knee joint area. According to clinical experiences, primary evidence of OA, like the joint space narrowing, appear on both sides of a knee. However, spatially distant feature extraction is challenging for a traditional CNN [13], of which convolutional filters only receive the information from a local region. As a result, the extracted feature maps do not address the relationship between different local regions. Researchers designed new convolution operators in the computer vision domain; for example, [14] proposed the dilated convolution. For OA diagnosis, Tuplin et al. divided the knee joint areas into the left and right sides [15]. Then, the authors used two CNNs to extract the features separately and fused them for classification.

Recently, [16] proposed the visual transformer, which takes advantage of relations between different local regions to boost the performance on multiple visual tasks. Transformer [17] was first applied to the natural language procession (NLP) field based on the self-attention mechanism. In the implementation, inputs are first encoded into three components: the query, the key, and the value. Then, the value is weighted by a mask calculated from the query and the key as in

(5) $$\begin{array}{c} \text{Attention}\left(Q,K,V\right)=\text{softmax}\left(\frac{Q\cdot K^{T}}{\sqrt{d_{k}}}\right)\cdot V, \end{array}$$

where *Q*, *K*, and *V* denote the query, key, and value components. And *d*_*k*_ is the dimension of key components. For an NLP task, *Q*, *K*, and *V* are the sequences of feature vectors extracted from each word in a sentence. The dot product of *Q* and *K* calculates the correlations between each pair of words in the sentence. Then, the softmax function normalizes the correlation and applies it to *V* as attention weights. In this case, only the features of the highly related words are emphasized. For a visual task, [16] took advantage of the self-attention mechanism and proposed the visual transformer. Images were divided into patches and reorganized into a sequence. Equation (5) uncovers the relationship between each pair of patches by calculating the correlation, even if the two patches are distant in the original image. Additionally, in [16, 17], the authors applied the “multihead” to the self-attention mechanism. The multihead technique contains multiple parallel self-attention layers, enhancing the capability to exploit more specific locations simultaneously.

## 3. Method

### 3.1. Data Preprocessing

Data used in this article was obtained from the Osteoarthritis Initiative (OAI) database, which is available for public access at http://www.oai.ucsf.edu/. Specific datasets used are 0.C.2 and 0.E.1.

The original dataset contains 16-bit DICOM X-ray files and assessment information of 4796 samples. They are collected from over 431,000 clinical and imaging visits. All X-ray files are converted to standard 8-bit gray-scale images using the Pydicom toolkit [18]. Most of the assessments by different annotators in the dataset are consistent. We rejected ambiguous samples whose assessments vary from different visits. 4506 samples are remaining in total.

### 3.2. Knee Joint Area Detection

The YOLO models demonstrate higher efficiency and speed on the objection tasks than the R-CNN series models [10]. Thus, we employ the YOLO model to tackle the issue of knee joint area detection. A valid knee joint segmentation, according to the radiologists, starts from the upper end of the tibia to the lower end of the femur, with the cartilage part lying at the center of the image. Parts of the fibula can be within this range. Following this standard, we use a Python-based tool [19] to annotate samples. To minimize the human efforts, we restrict the number of labeled samples to be 200. It accounts for 4.43% of the whole dataset.

The original YOLO architecture is modified to adapt to the knee detection task. As discussed in the previous section, the bounding box regression requires five outputs from the model per prediction per anchor. The total output channels can be calculated as *B* × (*C*+5), where *B* is the number of anchors and *C* is the number of object class labels. The original model uses five anchors and is trained on the COCO dataset [20], which contains 80 class labels. Thus, it has 5 × (5+80) channels in the last convolution layer. The only label to be predicted in the knee detection task is the “knee joint,” which determines the number of channels in the last layer as 5 × (1+5)=30.

Fine-tuning faces two challenges: (1) the number of annotated samples is limited and (2) the model validation is difficult as there is no ground truth for the testing data. In our implementation, we use transfer learning to overcome the difficulty caused by insufficient data. Except for the final layer, initial weights are obtained from the pretraining on the COCO dataset [20]. In addition, the training uses all annotated samples. Meanwhile, we monitor the intersection over the union (IOU) score defined in

(6) $$\begin{array}{c} \text{IOU}=\frac{A\cap B}{A\cup B}, \end{array}$$

where *A* denotes the predicted bounding box and *B* denotes the ground truth. Once the IOU scores converge, the training is terminated to avoid overfitting. Then, the YOLO model predicts the bounding boxes of the rest of the 95.57% of images. Unlike the typical validation process, the segmentation results are verified by statistical analysis discussed in the next section.

### 3.3. KL Level Classification

The severity of OA is categorized by the Kellgren–Lawrence (KL) grading system, which contains five levels ranging from KL-0 to KL-4, as shown in Table 1. The KL-0 grade represents that no radiographic evidence of osteoarthritis is present. In contrast, KL-4 indicates the latest stage of OA containing severe joint space narrowing and sclerosis.

Following the knee detection, ROIs are cropped according to the predicted bounding boxes. Before the classification task, each image is resized to 224 × 224 and normalized by the mean and variance computed from the training data. Preprocessing is one of the data-based interpretation strategies used for transfer learning [21]. Resizing and normalization adjust the statistical properties of the knee images to match the data used for pretraining. In [22], the author also employed a similar technique to handle knee ROIs.

The classification process has three steps, as shown in Figure 2.

Firstly, a CNN backbone extracts the spatial features from the knee ROI images. In our implementation, the CNN backbone is based on the ResNet50 [11] architecture, where the last pooling and dense layers are removed. The output of the backbone is denoted as *O*^(*C* × *H* × *W*)^, where *C*, *H*, *W* are the numbers of channels, height, and width. Given an image of 224 × 224, the output of the ResNet50 backbone is *O*^(1024 × 14 × 14)^. Notably, spatial feature maps preserve the extracted features from different local regions. As illustrated in Figure 2, the first feature vector contains the features from the corresponding top left corner region of the knee images.

Secondly, the spatial feature maps are flattened and combined with class label tokens and position embedding. As the size of each feature map is 14 × 14, it corresponds to 196 local regions of the original image. By reshaping *O*^1024×14×14^ to 196 × 1024, we rearrange the feature vectors into a matrix *M*, where each row contains the features from the same region.

Thirdly, the visual transformer exploits the relationship of the features from different regions. The visual transformer block follows [16], which contains twelve parallel self-attention layers. Each self-attention layer consists of two parts: (a) a self-attention block: as discussed in the previous section, the self-attention block projects inputs into *K*, *Q*, *V* and the weighted features are calculated by equation (5) and (b) a two-layer neural network: followed by the self-attention block, the two-layer neural network processes the features and sends them to the next transformer block. Both of the above two parts have a residual connection, which adds the inputs to the outputs [11]. In total, the proposed method uses 12 visual transformer blocks followed by a dense layer for the OA severity classification.

## 4. Experiment Results and Discussion

### 4.1. Knee Area Segmentation

The YOLO model was trained with darknet [23] for 3000 iterations. The batch size and optimizer settings were the same as the original work.  Figure 3 shows the IOU score of each training batch. The moving average IOU scores over 50 batches were used as the indicator of convergences. After training, the IOU score on the annotated 200 samples reached 0.82.

Figure 4 shows four examples of the detection results on the remaining samples. However, the IOU score is unsuitable for verifying knee detection because the remaining samples do not have annotations. To validate the segmentation results, we proposed four statistical forms of measurements.

1. Detection count per image: thanks to the consistency of the OAI dataset, all collected screen data consist of two knees. Therefore, two detections per image are expected.
2. Detection size: the sizes of the knee are similar for humans. However, knee detection varies due to the scale of the X-ray image. From the statistical view, the detections are expected to tend to cluster.
3. Detection location: a proper pair of knee joint detections should be located on the same height vertically and on both sides of the image horizontally.
4. Object confidence: as all images contain the knee joints, a reliable model should give a high confidence score on its detection.

From the four aspects mentioned above, we evaluate the detection results from the testing images. Firstly, Figure 5 shows the distribution of detection per image. 98.22% of images in the dataset have two detections corresponding to the left and right legs. The YOLO model successfully detects two knees in most images. Secondly, Figures 6(a) and 6(b) show the distributions of height and width for both original X-ray images and cropped ROIs. As shown in Figure 6(a), the sizes of the original X-ray images are separated into two clusters. The centroids of the two clusters are located near (600,500) and (1100,850). Correspondingly, Figure 6(b) shows two clusters regarding the sizes of the cropped ROIs, whose centroids are near (150,125) and (250,200). The clustering of cropped ROIs can be explained by the scale of original X-ray images, as the knees area is in proportion to the X-ray image size. Therefore, the sizes of detected ROIs are comparable. Moreover, the results also demonstrate that the trained YOLO model is robust to different X-ray image sizes.

Thirdly, Figure 7 shows the locations of all detected knees, which are represented by the top-left corner's coordinates. We observe two groups of detections marked as “X” and “Y.” The centroids of group “X” lie near (150,200) and (400,200). Regarding the ROIs in group “Y,” their y-coordinates range between 280 and 400, and their x-coordinates are near 200 and 600. Vertically, all detections appear in the middle region of the X-ray image. Horizontally, the clusters distribute on the left and right sides.

Finally, Figure 8 shows the confidence score distribution and the Kernel density estimation line based on the scores given by the YOLO. The center of the score distribution is roughly 85%. It indicates that the trained model has high confidence in its prediction.

Based on the above four measurements, we can conclude that segmentations on the whole dataset are accurate and valid. Furthermore, to mitigate the influence of invalid detections, we use the confidence score of 0.75 as a threshold to filter the ROIs referring to the predicted confidence score. In this way, we preserve 95% of ROIs, and their label distribution is shown in Table 2.

As shown in Figure 4, the YOLO model locates the knee joint areas which are used by radiologists to diagnose OA. Irrelevant bones and muscles were removed after we cropped the image according to the detected bounding boxes. The object detection CNN reduces the cost of manual feature selection, which resolves the challenge of noise elimination mentioned in Section 1

### 4.2. Classification Result

For the classification task, obtained ROIs were split into training set and validation set by the ratio of 8 : 2. The KL label distribution is shown in Table 2. We used the same augmentation method for the training set as in [22] to slightly adjust the brightness and contrast. For optimizer, we used the Adam with a learning rate of 1*e *−* *4 and the weight decay of 1*e *−* *8. Similar to [15], all models in our experiment were initialized with the pretraining weights from the ImageNet dataset [24]. We did not use a learning rate scheduler in our work. The metric used for the classification is the accuracy score over five KL grades. We ran the ResNet50 and ResNet101 as the baseline. Besides, the results were compared to the accuracy reported by recent studies on the same OAI dataset, including [15, 22, 25]. The accuracy scores are shown in Table 3.

Compared to the baseline ResNet50, the proposed method makes a 2.5% improvement. As discussed in the last section, traditional CNN has difficulty fusing the features from different local regions. When we use ResNet101, the improvement is trivial, implying that the depth of the network is not the bottleneck of performance. The results obtained from [22] have the same trends that the performance of ResNet101 is lower than ResNet50. On the contrary, the newly added visual transformer blocks consider the relationship between different local regions. Through the self-attention mechanism, features from key regions are emphasized, which helps improve classification performance.

To illustrate the attention maps, we randomly choose five samples from the validation set and draw the attention maps for the ResNet50 and the proposed method. For ResNet50, we use GradCAM [26] to show the activated areas which support the model's classification results. For the proposed method, we employed the attention flow technique [27] to extract the attention weights from the visual transformer.  Figure 9 shows the attention maps over the X-ray images where the images in the top row are the results of ResNet50, and the bottom row is the result of the proposed method. Regions highlighted by red color have higher weights when supporting the CNN to make a decision. As shown in the top row, ResNet50 succeeds in capturing the knee joint areas, which are the major lesion of knee OA. However, attention maps of the proposed method differ from ResNet50 in two aspects. Firstly, the attention map of ResNet50 shows only one centralized high attention region, which is either in the middle or on one side of X-ray images. On the contrary, the high-weighted areas spread out on both sides of the X-ray images. As discussed in Section 3.3, the visual transformer explores the correlation between small regions. As shown in Figure 9(f), the proposed method takes advantage of the correlation between both sides of the bone and shows superior performance in locating the narrow joint spaces. Secondly, ResNet50 can hardly detect sclerosis or bone spurs outside the knee joint areas. Through fine-grained region division, the proposed method detected the lesion areas on the medial or lateral edge of the femur as in Figures 9(f)–9(j).

During the course of writing this paper, we noticed that the authors in [22] employ a similar way for knee segmentation. However, unlike the method proposed by [22], we enhance the model performance from a different angle. In [22], the authors focused on the loss function. They designed an ordinal loss to identify the ambiguous samples of adjacent KL grades. The proposed method solves the classification task by enhancing the feature extraction. Despite the competitive results of [22], we still outperform them using the same ResNet50 backbone.

Merging the features from different regions to assess OA is firstly explored by [15]. The authors used a Siamese net containing two CNNs to extract features from both sides of the knee. Before feeding into the CNNs, knee images were vertically divided into two parts from the center. Then, two CNNs processed images independently. In addition, feature vectors were concatenated into one for the final classification. The image separation was based on the medical experience. The authors also conducted the experiments based on the dataset from multiple sources. As only two regions were considered in [15], the granularity of the region can be enhanced further. Thanks to the visual transformer, we exploit the relationship of more fine-grained local regions. In addition, the fusing of the features is automatic and learnable. As a result, our method improves the performance of the OAI dataset.

## 5. Conclusion

In this paper, we presented a highly automatic process to diagnose osteoarthritis based on deep learning. We demonstrated that transfer learning from the object detection domain could be successfully applied to knee joint area segmentation. A model trained on 4.43% of annotated data can extract accurate ROIs on the remaining data, containing more than 4500 samples. For the OA severity classification, we employed the visual transformer to exploit the correlations between different regions of the original X-ray image. Experiment results show that the proposed method improves the OA severity classification performance compared to the previous state-of-the-art methods. The following aspects distinguish our approach from previous ones.

1. Human efforts on preprocessing raw radiographic images are reduced to a negligible level.
2. The segmentation procedure is highly automatic. As shown in the segmentation results, the reliability and accuracy of the segmentation outcomes demonstrate the reusability of our trained model.
3. Taking advantage of the self-attention mechanism, the visual transformer blocks built on top of traditional CNN architecture improve the classification performance.
4. Once built, the proposed procedure is an end-to-end solution to OA diagnosis. Raw X-ray images can be sent into our pipeline directly. All adjustments are handled internally, such as resizing and enhancing.

We notice that our experiment is conducted on the dataset from a single vendor. In the future, we would like to explore the application of our method on the data from multiple sources.

## Figures and Tables

**Figure 1:** Computer-aided OA diagnosis pipeline. The entire process consists of two stages, including knee segmentation and OA severity classification. Typically, the knee segmentation depends on human efforts or manually selected features. Then, a machine learning model, such as CNN, is trained to classify the knees based on the OA severity grades.

**Figure 2:** Overview of the proposed method. The OA severity assessment is divided into four steps. (1) An object detection CNN extracts the bonding boxes of the knees from the X-ray images. The confidence scores of the detection are used to filter the low-quality detection. (2) A CNN backbone extracts the spatial feature maps for the cropped knee images. (3) The spatial feature maps are flatted and recomposed as a sequence. (4) The visual transformer exploits the correlations between different local regions for the final classification task.

**Figure 3:** The IOU score for each batch (iteration) during training. The moving average value of 50 batches is marked as “50-Batch Ave. IOU” to show the general trend.

**Figure 4:** Automatic segmentation examples.

**Figure 5:** Detection count per image. In total, 4426 images have 2 detections, which account for 98.22% of the whole dataset.

**Figure 6:** Size of the original images and detections. (a) The size of original image. The OAI dataset has two clusters of shapes, as indicated in the red and blue colors. (b) The knee segmentation widths and heights. Two clusters regarding the size of the bounding box are marked by red and blue, respectively.

**Figure 7:** Locations of knee detections. Vertically, all detections appear in the middle region of the image except for outliers. Horizontally, two pairs of clusters are labeled as “X” and “Y” according to the positions. The clusters are caused by different X-ray image sizes and knee alignment. Cluster “X” has only one pair of centroids. While cluster “Y” is split into 3 subgroups. Each subgroup on the right has its counterpart on the left.

**Figure 8:** Object confidence score distribution (by the YOLO model). The distribution of confidence scores is centered at 85. The density of low confidence detection (below 75) is nearly zero. The confidence score distribution indicates that the majority of detections are reliable.

**Figure 9:** Comparisons of the attention maps of ResNet50 and the proposed method. The first row (Figure (a) to Figure (e)) shows the activated areas of the ResNet50 model generated by GradCAM. The second row (Figure (f) to Figure (j)) shows the attention weights of the visual transformer extracted through the attention flow technique. For each column, input X-ray images are the same. The proposed method succeeds in locating the narrow joint spaces on both sides of the knee. In addition, we detect sclerosis or bone spurs on the medial or lateral edge of the femur as in (f), (g), and (j).

**Table 1:** Definition of the Kellgren–Lawrence grading system.

Grade	Remarks

KL-0	No evidence of osteophyte
KL-1	Doubtful osteophyte
KL-2	Definite osteophyte; possible joint space narrow (JSN)
KL-3	Moderate osteophytes, definite JSN, some sclerosis, and possible deformity of bone ends
KL-4	Large osteophytes, definite JSN, sclerosis, and deformity of bone ends

**Table 2:** Label distribution of the cropped ROI.

	KL-0	KL-1	KL-2	KL-3	KL-4
Total ROI	3234	1475	2186	1141	266
Training set	2587	1180	1749	913	213
Validation set	647	295	437	228	53

**Table 3:** Comparisons of classification results.

Model	Accuracy (%)
VGG-19 [25]	53.4
ResNet50	66.68
ResNet101	66.70
Ordinal loss (ResNet50) [22]	66.2
Ordinal loss (ResNet101) [22]	65.5
Siamese net [15]	66.71
The proposed method	69.18

## Data Availability

Data used in the preparation of this article were obtained from the Osteoarthritis Initiative (OAI) database, which is available for public access at http://www.oai.ucsf.edu/. Specific datasets used are 0.C.2 and 0.E.1.
